RETRACTED

# Value Analysis of Using Urinary Microalbumin in Artificial Intelligence Medical Institutions to Detect Early Renal Damage in Diabetes

**DOI:** 10.1155/2021/6678454

**Published:** 2021-03-12

**Authors:** Sitong Lin, Yushan Guo

**Affiliations:** Department of Endocrinology, Affiliated Hospital of Beihua University, Jilin 132012, China

## Abstract

As the scale and depth of artificial intelligence network models continue to increase, their accuracy in albumin recognition tasks has increased rapidly. However, today's small medical datasets are the main reason for the poor recognition of artificial intelligence techniques in this area. The sample size in this article is based on the data analysis and research on urine albumin detection of diabetes in the EI database. It is assumed that the observation group has at least 20 mg UAER difference from the control group, and the standard deviation of the UAER change from baseline to 12 weeks is 30 mg. Therefore, the sample size of the two groups is 77 cases. Assuming that the rate of loss to follow-up during the follow-up period is 20%, at least 92 patients are needed. The final enrollment in this study is 100 patients. Studies have shown that DR is used as an indicator to diagnose NDRD, and its OR value is as high as 28.198, indicating that non-DR can be used as an indicator to distinguish DN from NDRD. The meta-analysis found that DR has a sensitivity of 0.65 and a specificity of 0.75 in distinguishing DN from NDRD in patients with type 2 diabetes, and it is emphasized that PDR is highly specific in the diagnosis of DN. Using a meta-analysis to systematically analyze 45 studies, it was found that the sensitivity of DR to diagnose DN was 0.67, the specificity was 0.78, and the specificity of PDR to predict DN was 0.99, indicating that DR is a good indicator for predicting DN, and the team's latest research has also verified this point of view. They have established a new model for diagnosing DN. In addition to including traditional proteinuria, glycosylated hemoglobin, FR, blood pressure, and other indicators into the diagnostic model, it will also include the presence or absence of DR. The final external verification accuracy rate of this model is 0.875.

## 1. Introduction

With the continuous development of proteomics, the proteomics technology system based on protein separation technology, biological mass spectrometry technology, protein interaction technology, and bioinformatics technology has solved the difficulty of accurately characterizing the proteome expression profile and is the DKD (diabetic kidney disease) research system establishment, and improvement of DKD provided technical support and laid a good foundation for DKD functional proteomics research. But there are still many shortcomings in urine albumin detection, which seriously affects the recognition of diabetes [1].

RETRACTED

Knobel used iTRAQ technology to identify potential urine biomarkers and verified them with ELISA. The results showed that haptoglobin (HPT) as a biomarker with significant content differences can distinguish healthy individuals from DKD patients [2]. Mise et al. used HPT as a candidate biomarker and evaluated the ability of haptoglobin/creatinine (HCR) to predict end-stage renal disease in DKD patients in Taiwan. The data indicated that HCR may be a ratio of urine albumin/creatinine (UACR) which is a more sensitive clinical evaluation index for predicting the progression of DKD [3]. Based on LC-MS/MS and random forest (rRF) algorithms, An et al. distinguish the urine peptide profiles of patients with DKD at different stages of type 2 diabetes [4]. Kimura collected and tested the urine of type 2 diabetic patients with different conditions, using bioinformatics methods, and first-ranked the important peptides in the DKD environment [5]. According to the course of diabetes and the severity of kidney damage [6], Maratos-Flier used a grouping strategy to analyze the urine proteome of samples by 2-DE and constructed a low MW (LMW) proteome map with a molecular weight (MW) <50 kD [7].

Groop PH screened 8 kinds of LMW proteins unique to diabetic patients, using these proteins, then analyzed the urine peptide sequence to predict the proteolytic characteristics associated with DKD, and explore the differential regulation mechanism of inflammation and complement system in DKD [8]. Hwang characterized the proteins in human urinary exosomes through LC-MS technology and found that the proteome in the DKD group and the healthy control group had significantly different levels of expression [9]. Dantas et al. analyzed the kidney tissue proteins of early DKD rats and found that calmodulin (CaM) and senescence marker protein (SMP) were significantly downregulated compared with healthy controls [10]. Lippi et al. used ESI-Q-TOF MS/MS technology to screen and found proteins that were significantly upregulated and downregulated in the development stage of DKD compared with control samples [11]. Viswanathan believes that autophagy is the main cell clearance mechanism for maintaining cell survival and homeostasis, and it plays an important role in the development of diabetes and DKD [12].

In order to evaluate whether urine exosomes can reflect changes that occur at the tissue level, this paper collected exosomes in urine samples. The study found that the proteome of exosomes and the proteome of kidney tissue have the same changing trend. This paper proposes an artificial intelligence-based diagnostic model for diabetic albumin membrane lesions. First, the collected albumin is analyzed, and the analyzed albumin is subjected to background removal, denoising, and normalization using a digital albumin processing algorithm. The protein pretreatment operation reduces the influence of albumin quality on the model training results; at the same time, in order to avoid the phenomenon of network model overfitting due to the small amount of albumin membrane albumin data, it is necessary to expand the data of the pretreated albumin and then load the processed data set into the deep convolutional neural network model for training. After training, the model can automatically detect the lesion level of the patient's albumin membrane albumin. The artificial intelligence algorithm is used to automatically extract the characteristics of albumin, and the traditional support vector machine (SVM), K nearest neighbor algorithm, and other steps that require feature detection and manual feature extraction of albumin are discarded, reducing human factors. The phenomenon of misdiagnosis can also greatly shorten the diagnosis time of diabetes, which is of great significance for the early prevention and treatment of patients with diabetes.

RETRACTED

## 2. Artificial Intelligence and Diabetic Kidney Disease

### 2.1. Artificial Intelligence Urine Microalbumin Detection Technology

The emergence of urine microalbumin detection technology has further improved the efficiency and accuracy of screening and identification of DKD (diabetic kidney disease) biomarkers and improved the characterization of the body's proteome expression profile in the DKD state. In order to explore the pathogenesis of DKD, screening early diagnostic markers and therapeutic targets and revealing the complex molecular regulatory network of DKD laid the foundation. The difference in protein expression levels predicts protein molecules closely related to diseases and verifies their functions to confirm target molecules related to diseases [13]. The primary task of DKD proteomics research is to construct and improve the research system, and its workflow mainly includes the separation, identification, and quantification of protein samples [14]. Common protein separation techniques can be divided into two methods: gel-based and nongel. Among them, gel-based technologies include 2-DE and 2D-DIGE. 2-DE technology is the core technology for separating proteins based on gels. The 2-DE can be used to separate hundreds of proteins on a single gel. It has the characteristics of high throughput and high resolution and can be used in conjunction with MS. Therefore, this technology has been widely used in comparative proteomics [15]. However, the traditional 2-DE technology has also certain limitations, such as poor reproducibility, difficulty to detect low-abundance proteins, and complex sample processing procedures that easily lead to protein loss. Therefore, the 2D-DIGE technology came into being [16]. Based on 2-DE, 2D-DIGE must perform different fluorescent labels on different protein samples prior to protein electrophoresis separation to complete a one-time electrophoresis separation of mixed samples. This technology realizes that the protein samples of different experimental groups are in the same block. Not only does a separation in the gel avoid the problem of poor 2-DE repeatability, but also the introduction of fluorescent internal standards can accurately detect the difference in protein abundance between different samples and significantly improve the accuracy and sensitivity of protein separation [17].

RETRACTED

However, for the separation and characterization of protein complexes, the above techniques are not applicable. This is because the harsh denaturation conditions can easily cause the dissociation or even denaturation of protein complex subunits, which makes it impossible to obtain a complete protein complex [18]. In contrast, nondenaturing electrophoresis technology provides a better choice, such as BN-PAGE and its derivatives CN-PAGE and hrCN-PAGE. The technical point is to introduce a bright blue dye with negative ions in the cathode buffer (CBB) or the anionic detergent sodium deoxycholate (DOC), which makes the surface of protein complexes carry a large number of negative charges during electrophoresis, which can not only prevent nonspecific aggregation between protein complexes but also increase the hydrophobic protein solubility, which improves the electrophoresis efficiency of protein complex samples; at the same time, a large number of negative charges on the surface can eliminate the difference in the charge of the protein complex itself, so that the mobility of the complex in the gel is only determined by its molecular weight (volume), which improves the electrophoresis resolution. Although BN-PAGE, CN-PAGE, and hrCN-PAGE techniques have been widely used in the separation and analysis of membrane protein complexes, the introduction of additional anions has an unavoidable impact on the gentle characteristics of electrophoresis and cannot be fully applied to weakly interacting protein complexes [19]. Based on this, the 4-DES and BS4-DES technologies derived from 2-DE, while taking into account the high resolution and gentle separation characteristics of BN-PAGE and hrCN-PAGE, break through the compatibility of diluted samples and the compatibility of basic proteins. The isoelectric point (pI) has a narrow separation range [20]. The main feature of the above two techniques is the addition of a two-dimensional nondenatured electrophoresis method before the conventional 2-DE modified electrophoresis including one-dimensional electrophoresis (1st-DE). Among them, IEF can achieve sample concentration and enrichment under mild nondenaturing conditions [21]. The second-dimensional electrophoresis of BS4-DES derived from 4-DES uses mild acidic and alkaline nondenaturing gel electrophoresis (PAGE) technology to extend the application range of protein p I to ∼3.0 to 11.0, which can smoothly realize the electrophoresis of alkaline sample separation [22]. Although the operation steps are more complicated than traditional 2-DE, while maintaining the advantages of 2-DE, 1st-/2nd-DE can maximize the integrity of protein complexes or interacting proteins, which is conducive to the subsequent first three- and four-dimensional electrophoresis (3rd-/4th-DE) which further explores more complex protein interaction information [23]. In addition to gel technology, the improvement and maturity of the above-mentioned protein separation technology have improved the proteome separation ability and reduced the impact of separation operations on the protein molecular structure. This is to solve the problem of the wide variety and different properties of proteins in the proteome of DKD patient samples. The difficulty of separation provides technical support and makes it possible to systematically complete the separation and analysis of the DKD proteome [24].

RETRACTED

### 2.2. Artificial Intelligence Protein Identification Technology

The identification work after protein separation can determine the type of protein in the sample, which is a key step in proteome analysis. In recent years, biological mass spectrometry technology has rapidly developed into a proteomic research technology for identifying high-throughput biological macromolecules. The soft ionization method can ensure that biological macromolecules will not produce too many fragment ions, which greatly simplify the complexity of the spectrum, which is conducive to subsequent further analysis [25]. ESI-MS is one of the main methods of protein identification. It is characterized by the easy generation of multicharged ions and fewer fragment ions. The formed ions can be directly used to determine the molecular weight of proteins or peptides with high sensitivity and multicharged ions. The formation of M/z significantly reduces the m/z value, so that ESI-MS can accurately determine large molecular weight proteins in a more suitable m/z detection range. MALDI-MS is another well-developed protein identification technology, often equipped with a time-of-flight (TOF) mass analyzer. This technology does not require complex preprocessing of protein samples, and the ionization of the molecule to be tested can be achieved through matrix assistance; fewer fragment ions are generated during the ionization process, and high-throughput rapid scanning of protein-peptide molecules can be performed to produce proteins. Peptide fingerprinting (PMF) combined with search engines (such as MASCOT) and specific databases (such as SwissProt and NCBInr) can complete protein search matching and identification [26]. In the case of unsuccessful PMF matching or low matching specificity, a joint search can be further combined with MS/MS secondary spectra to achieve accurate multidimensional analysis and identification of proteins. Up to now, in addition to biological mass spectrometry identification technology, choosing a suitable protein identification strategy is also the key to protein identification work [27]. With the rapid development of the above-mentioned biological mass spectrometry technology, the main strategies of protein identification can be summarized as follows: bottom-up (BU), middle-down (MD), and top-down (TD) strategies. The so-called bottom generally refers to peptides, top refers to the complete protein, up refers to the inference process from peptide to protein, and down refers to the process of fragmenting the complete protein molecule through tandem mass spectrometry. In the BU strategy, the shotgun-based proteomic multidimensional chromatography-biomass spectrometry identification method is one of the most important research methods [28]. Its disadvantage is a large amount of data, the complexity, and difficulty of data analysis, and the peptide is the protein sequence coverage rate identified by the center which is very low, less than 20%, and the enzyme digestion process will cause the loss of important information such as PTMs, which hinders the accurate functional analysis of the protein. In response to the shortcoming of the BU strategy that protein PTMs are easy to lose, MD strategy came into being. This technology uses biological enzymes different from the BU strategy to obtain as many longer peptides with PTMs as possible, so that subsequent mass spectrometry analysis can be more comprehensive and accurately characterize the fine structure of the protein. The TD strategy does not require protein digestion. Based on maintaining the integrity of the protein structure, it first performs a molecular contour scan (such as molecular weight) and then uses a variety of cleavage techniques such as collision induction/activated cleavage (CID/CAD). Up to now, the pathogenic mechanism of DKD has not been clearly elucidated, and the sensitivity and accuracy of commonly used clinical diagnostic methods are not very satisfactory, which makes the determination of the treatment plan after DKD diagnosis more difficult than general kidney disease. As the main undertaker and embodiment of life activities, protein directly participates in and regulates various life processes. Carrying out DKD research from the proteomics level can explore the relevant molecular mechanisms of the disease from the perspectives of overall, dynamic, and interactive networks. Proteomics research on DKD clinical samples under different physiological and pathological conditions can comprehensively explore the key proteins that are significantly related to DKD; through in-depth analysis and verification of these proteins, we can more intuitively understand the molecular mechanism of DKD development, and obtaining candidate markers related to the DKD process and potential therapeutic targets for subsequent diseases will lay the foundation for the early diagnosis of DKD and the exploration of new treatment methods. In recent years, with the continuous development of proteomics technology, many emerging technologies have been derived from the core proteomics technologies such as protein separation, mass spectrometry identification, and bioinformatics analysis, which have further promoted proteomics in disease biomarkers screening, revealing the molecular mechanism of pathogenicity, and the application of drug action protein targets. Based on proteomics research technology, this article mainly reviews the application progress of proteomics in DKD research from three aspects: research on the pathogenic mechanism of DKD, screening of potential biomarkers for early diagnosis, therapeutic targets, and effect evaluation. Although proteomics has made great progress in DKD research, it still has a large room for development, especially the correlation analysis of a large number of potential DKD molecular markers that have been identified, the clinical verification and application of drug-protein targets. It is the focus of DKD's future research. In areas with a high incidence of urinary disease, the current early diagnosis of DKD is relatively poor, leading to a partial missed diagnosis of early disease patients, which is difficult to reverse when diagnosed. At the same time, a large number of domestic and foreign scholars have conducted in-depth research on the molecular mechanism of the pathogenesis, pathogenesis, and treatment of DKD. Studies have shown that pathogenic factors such as hyperglycemia, hypertension, hyperlipidemia, and hemodynamic changes are all involved in the occurrence and development of DKD. At present, it is generally believed that DKD is a complication induced by the body being in a long-term unhealthy state. It is difficult to fully explain the dynamic regulation process of the patient's internal environment on the development of the disease from a genomics level. Therefore, it is necessary to further promote DKD from a new perspective. Up to now, DKD has been studied in depth on the overall level. Among them, transcriptomics mainly studies the transcription level of related genes at different stages of DKD, the regulation of transcription, and the search for biomarkers for early diagnosis of diabetic nephropathy, risk prediction, and prognosis judgment [29]. Proteomics is a comprehensive and in-depth study of the proteome of tissue cells and body fluids such as blood, urine, and saliva of DKD patients to characterize DKD protein expression profiles and screen key DKD protein biomarkers. As the main undertaker and executor of life functions, protein can most directly reflect biological characteristics. Proteomes are highly diverse, complex, and highly modified and are specific to tissues and cells, and their expression levels, structures, and functions vary depending on regulations. Therefore, proteomics can reflect the dynamic changes of the body's protein levels in pathological conditions by detecting the proteome expression of tissue samples at a specific time and more intuitively explain the molecules of DKD from the perspective of the overall, dynamic, and interactive network. This mechanism deepens people's understanding of complex diseases and provides new ideas for the prevention, diagnosis, and treatment of DKD. In disease proteomics research, proteomics technology is mainly used to study the differential expression of proteins in various patient samples at different periods and different physiological states and to fully characterize various physical and chemical properties of proteins in disease states, including expression level, structure, distribution, function, and posttranslational modifications (PTMs), to analyze the interaction between proteins and between proteins and diseases, and to construct protein molecular networks in disease states.

RETRACTED

### 2.3. Artificial Intelligence Model for Extracting Lesion Features of Diabetic Albumin

*Artificial Intelligence Model Performance Evaluation Index*. In order to quantitatively compare and analyze the classification results of recognition networks, this paper uses two indicators of model accuracy and space complexity to objectively evaluate the classification effects of various recognition networks. The indicators used to evaluate the classification effect of the model include accuracy and average accuracy. The calculation formulas are as follows:

(1) $$\begin{array}{c} E=\frac{\sum_{j=1}^{k}\sum_{h=1}^{k}\sum_{t=1}^{n_{j}}\sum_{r=1}^{n_{h}}\left|y_{ij}-y_{hr}\right|}{2n^{2}u}, \end{array}$$

where *E* represents the number of samples correctly classified and *K* represents the number of samples tested. The activation function has a slope gradient of 1 for all positive inputs, indicating that using the IC activation function can make the gradient descent run faster and effectively reduce the training time.

(2) $$\begin{array}{c} I_{A}=E_{w}+E_{nb}+E_{t}-Ic. \end{array}$$

In the DetectionNet model structure proposed in this article, different convolutional layers use multiple convolution kernels to extract diabetic albumin lesion features:

(3) $$\begin{array}{c} SC=\left(P\times Q\right)-1,\\ E_{j}=\frac{\left(1/2u_{j}\right)\sum_{i=1}^{n_{j}}\sum_{r=1}^{n_{j}}\left|y_{ji}-y_{jr}\right|}{n_{j}^{2}},\\ Ew=\sum_{j=1}^{k}G_{jj}p_{j}s_{j}. \end{array}$$

In addition, albumin has rich detailed features. If the convolution field of view is too large, it is not conducive to the extraction of detailed features. The convolutional neural network in this article uses two 3 x 3 convolutions to replace a 5 x 5 convolution in the *E*_*w*_ module:

(4) $$\begin{array}{c} I_{B}=\frac{\sum_{Z=1}^{h_{j}}\sum_{r=1}^{n_{h}}\left|y_{ji}-y_{hr}\right|}{n_{j}n_{h}\left(u_{j}+u_{h}\right)},\\ E_{nb}=\overset{k}{\underset{j=2}{\sum }}\overset{j-1}{\underset{h=1}{\sum }}G_{jh}\left(p_{j}s_{h}+p_{h}s_{j}\right)D_{jh},\\ E_{t}=\sum_{j=2}^{k}\sum_{h=1}^{j-1}G_{jh}\left(p_{j}s_{h}+p_{h}s_{j}\right)D_{jh}\left(1-D_{jh}\right). \end{array}$$

This paper uses the deep convolutional neural network DCNN as the training model for the identification of diabetic albumin membrane lesions. The training network model is based on Google's Inception albumin classification and recognition model, but albumin membrane disease albumin has its own characteristics. On this basis, it is necessary to adjust network parameters such as parameter setting and network model configuration to make it more suitable for classification training and recognition of albumin membrane lesions:

(5) $$\begin{array}{c} M=\frac{d_{jh}-P_{jh}}{d_{jh}+P_{jh}}. \end{array}$$

Even when the albumin is deformed or there is noise, it will not have a significant impact on the recognition results; on the other hand, it reduces the complexity of the network model and reduces the network parameters through the method of local perception field and shared weights, which is better than traditional models. Higher accuracy is as follows:

(6) $$\begin{array}{c} v\left(u_{i},p_{k}\right)=\frac{f\left(u_{i},p_{k}\right)\times \;\log\left(\left.m/mu_{i}\right.+0.01\right)}{\sqrt{\sum_{p_{k}}^{u_{i}}uf\left(u_{i},p_{k}\right)\times \;\log\left(\left.m/mu_{i}\right.+0.01\right)}}\times \text{const}\left(p_{k}\right),\\ d_{jh}=\int_{0}^{\infty }dF_{h}\left(y\right)\int_{0}^{y}\left(y-x\right)dF_{j}\left(y\right). \end{array}$$

Increasing the training data set is the most direct solution to overfitting the training model. However, due to the shortage of the data set, no additional data albumin can be provided. Therefore, it can be treated without changing the albumin disease level of the original data set. Perform operations such as zooming, rotating, flipping, and changing the brightness to make the albumin quantity of each disease level data set equal:

(7) $$\begin{array}{c} f\left(x\right)=\frac{1}{Nh}\sum_{i=1}^{N}k\left(\frac{X_{i}-x}{h}\right),\\ k\left(x\right)=\frac{1}{\sqrt{2\pi }}\exp\left(-\frac{x^{2}}{2}\right). \end{array}$$

After the data is expanded, the category with a larger number of samples has less impact, and the category with a smaller number is expanded to complement the category with a larger number:

(8) $$\begin{array}{c} h_{t}=\tan\;h\left(w_{c}x_{t}+u_{c}\left(r_{t}\Theta h_{t-1}\right)+b_{c}\right),\\ h_{t}=z_{t}\Theta h_{t-1}+\left(1-z_{t}\right)\Theta h_{t}. \end{array}$$

The loss function of this part includes two parts, the confidence loss and the category loss shown in

(9) $$\begin{array}{c} P=\sigma t=\frac{\sqrt{\left.1/n\right.\sum_{i=1}^{n}{\left(FI_{it}-FI_{it}\right)}^{2}}}{FI_{it}}, \end{array}$$

(10) $$\begin{array}{c} u_{\left(j\backslash i\right)}=w_{ij}A_{i}, \end{array}$$

A probability value *P* is assigned to this point, *P* is a random number between 0 and 1, and *P* is compared with the generation probability Prob; there are

(11) $$\begin{array}{c} \ln\left(\frac{PI_{it}}{PI_{it}-1}\right)=\alpha +\beta \;\ln\;PI_{it}-1+v_{i}+{ℑ}_{t}. \end{array}$$

The proposed loss function makes the bounding box regression process of target detection faster and more accurate than the previous loss function. The loss function is shown in

(12) $$\begin{array}{c} r=\frac{\alpha }{1-\beta }, \end{array}$$

(13) $$\begin{array}{c} \theta =-\frac{1}{T}\ln\left(1+\beta \right). \end{array}$$

Pathological identification has higher requirements for convolutional neural networks [30] and requires a deeper network to better fit the entire data set, and the expression ability of the model is stronger. However, in practice, as the network depth increases, there will be phenomena such as gradient disappearance and gradient explosion, resulting in a positive correlation between the depth of the network and the performance of the model.

RETRACTED

## 3. Urine Microalbumin Detection of Early Kidney Damage in Diabetes

### 3.1. Processing of Research Samples

The sample size in this article is based on the data analysis and research on urine albumin detection of diabetes in the EI database. The observation group has a UAER difference of at least 20 mg from the control group, and the standard deviation of UAER changes from baseline to 12 weeks is assumed to be 30 mg. Therefore, the sample size of the two groups is 77 cases. Assuming that the rate of loss to follow-up during follow-up is 20%, at least 92 patients are needed. A total of 100 cases were enrolled in this study. And after treatment, the UAER of the observation group decreased even more (*t* = 3.776, *P* < 0.001). After adjusting for age, gender, FPG, 2 h PPG, and HbA1c variables, the observation group UAER still showed a significant decrease (*F* = 24.60, *P* < 0.001).

### 3.2. Processing and Operation Steps

In order to explore the relationship between urinary microalbumin and early kidney damage in diabetes, this article uses artificial intelligence technology, 2-DE and MALDI-TOF-MS technology combined with the MASCOT search and identification engine to study long-term exposure to HG (high-glucose environment) condition protein expression profile of podocyte cell line. The identified differential proteins mainly belong to cytoskeleton proteins and specific annexins. The downregulated expression of annexin in glomeruli is also confirmed in patients with DKD. Annexin is a Ca2+ binding protein and phospholipid-binding protein involved in cell membrane organization and transport, and as a membrane scaffold, annexin also participates in the construction of a specific podocyte slit membrane. Therefore, the HG environment affects the construction of the podocyte slit diaphragm by downregulating the expression of annexin, destroys the glomerular filtration barrier, and induces the occurrence and development of DKD. In addition, this paper performed a proteomic integration network analysis on a large amount of relevant data obtained and used HG-treated distal renal tubular cells to conduct a variety of targeted function studies.

*The Application of Proteomics in the Study of the Pathogenesis of DKD*. Understanding the internal mechanism of the occurrence and development of DKD is very necessary for researchers to establish new diagnostic methods and develop new treatment ideas. The application of proteomics in the diabetic nephropathy process from diabetes to diabetic nephropathy involves a series of complex molecular regulation mechanisms. This article systematically analyzes biological samples of patients with DKD, revealing part of the pathogenesis of diabetic nephropathy, and in the early stage of DKD. Certain results have been achieved in diagnosis and treatment, which have promoted people's understanding of the occurrence, development, prediction, and remission of the disease and laid a good theoretical and experimental basis for the comprehensive treatment of DKD. In the DKD research, the establishment of a complete urine proteome database in this paper is the basis for the development of disease urine proteome research. This article attempts to define the urine proteome in various clinical settings, and through various proteomics methods, approximately 800 proteins have been identified, laying a foundation for candidate molecules for the discovery of biomarkers from the urine proteome.

RETRACTED

## 4. Urine Microalbumin Detection of Early Renal Damage in Diabetes

### 4.1. Artificial Intelligence Albumin Detection of Kidney Damage under Hierarchical Network

This article uses urine microalbumin samples to train the artificial intelligence model. As shown in Figure 1, although artificial intelligence neural network models are used to train the same data set, the accuracy of the training models is quite different, indicating that the neural network model structure directly affects the accuracy of the recognition results. LeNet has only an eight-layer network with the least space complexity and two convolutional layers suitable for extracting some simple albumin features. It is somewhat inadequate for the extraction of complex albumin features such as pathology.

As shown in Table 1, although the AlexNet network model is more complex, the increase in the depth of the network model will result in an increase in network parameters. If the training data is small, overfitting will often occur. The DetectionNet deep convolutional neural network designed in this paper is improved on the basis of the inception model. Under the premise of ensuring accuracy, the space complexity of the model is greatly reduced, which can not only accelerate the convergence speed of the model but also effectively avoid the occurrence of network congestion. The overfitting phenomenon is more suitable for the detection of diabetic albumin lesions.

As shown in Figure 2, while improving the detection function, a significant decrease in UAER was observed, further supporting the important effect of removing the albumin state in improving MA. At the same time, it was observed that insulin intensive hypoglycemia has a better effect of lowering MAU. At the same time, after correcting for age, gender, FPG, 2hPPG, and HbA1c confounding factors, it was found that diabetes treatment still showed a significant MAU reduction effect, which was compared with the diabetes treatment group blood sugar. The level of control is not significantly related.

RETRACTED

As shown in Table 2, for the diabetic albumin lesion grade diagnosis method, after the data set is normalized and after albumin preprocessing, data set expansion, and other data set preprocessing operations, the artificial neural network model is used to analyze the processed data. The data set is trained to generate a diabetic albumin lesion diagnosis model. Compared with other methods, the network model has a higher recognition rate and appropriate algorithm complexity. It can not only reduce the misdiagnosis caused by human factors but also greatly shorten the diagnosis time of diabetic albumin lesions. The early prevention and treatment of patients are of great significance.

The results of albumin detection and analysis are shown in Figure 3. The urine of DKD patients is similar to that of the elderly, and the correlation between biomarkers and aging and kidney disease has been confirmed. In addition, among healthy subjects, an age-related peptide excretion pattern was observed in the urine of some subjects. It is speculated that these people may have a higher risk of DKD. As shown in Table 3, DKD and kidney aging may have a common mechanism, which further explains that when looking for DKD biomarkers, the correlation between aging and kidney disease must be considered, and candidate biomarkers that can exclude the influence of age should be selected.

### 4.2. Mechanism Analysis of Albumin Aggregation and DKD in High-Glucose Environment

As shown in Figure 4, the HG environment can lead to the accumulation of intracellular protein, induce the accumulation of reactive oxygen species (ROS), lead to the imbalance of antioxidant homeostasis, interfere with energy balance, and cause Ca^2+^ absorption obstacles in distal renal tubular cells, which will eventually lead to renal tubules. As shown in Table 4, based on the targeted function study of integrated proteomic network analysis, this study confirmed the significant interference effect of the HG environment on the distal renal tubular cells, which helps to better understand the pathogenic mechanism of DKD.

As shown in Figure 5, DR can be used as an indicator for the diagnosis of NDRD, and its OR value is as high as 28.198, which indicates that non-DR can be used as an indicator for distinguishing DN from NDRD. The meta-analysis found that the sensitivity and specificity of DR in differentiating DN from NDRD in patients with type 2 diabetes mellitus were 0.65 and 0.75, respectively, and it was emphasized that PDR was highly specific in the diagnosis of DN. After systematic analysis of 45 studies by meta-analysis, it was found that the sensitivity of DR in the diagnosis of DN was 0.67, the specificity was 0.78, and the specificity of PDR in the prediction of DN was 0.99, suggesting that DR is a good indicator for the prediction of DN, and the latest research of the team also verified this view. They established a new model for the diagnosis of DN, in addition to the traditional proteinuria, glycosylated hemoglobin, FR, blood pressure, and so on. In addition to the indicators included in the diagnostic model, DR was also included. The final external validation accuracy of the model was 0.875. However, due to the limitation of renal biopsy requirements, the renal biopsy of clinical diabetic patients is not typical, and large sample studies are needed to verify and analyze the renal biopsy of diabetic patients.

RETRACTED

As shown in Figure 6, the etiology of DKD is very complex, and a variety of mechanisms are involved in the development of diabetic nephropathy. Protein is one of the main regulatory factors of cell physiology and ecology. Using proteomic methods to obtain qualitative and quantitative information on proteins will help to reveal the pathogenesis of diabetic complications. At present, the general strategy to analyze the pathogenesis of DKD from the level of proteomics is to use the comparative proteomics method to establish differential protein expression profiles between normal samples and DKD samples, in order to obtain DKD protein markers and to carry out biological function targeting research on the potential protein markers. DKD is a complex complication of diabetes. Abnormal expression of protein and signal pathway in diabetic patients exposed to a high-glucose environment (Hg) for a long time can easily lead to severe morphological changes of the kidney.

As shown in Figure 7, there are differences in physical function depending on the age group. Studying the influence of age on urine proteome is one of the factors that need to be considered comprehensively in screening and discovering relevant biomarkers. In this paper, the CE-MS method was used to analyze the low molecular weight proteinuria of healthy people of different ages. A total of 5000 kinds of urinary peptides were detected, among which 325 kinds of relative abundance were related to age. Most of these changes are related to kidney development before and after puberty. There are 49 kinds of polypeptides related to aging in adults.

As shown in Figure 8, the risk of CKD progression in patients with *R* is 16.6 times higher than that in patients without DR. It is worth noting that these studies all use proteinuria or EGFR to diagnose nephropathy but cannot make a clear diagnosis of DN, and many studies use ophthalmoscope or indirect ophthalmoscope instead of gold standard color photography for the diagnosis of DR at baseline. Therefore, although the correlation between PDR and DN can be made clear, the diagnostic value of PDR for DN still needs to be further studied. As shown in Table 5, the higher the UACR, the greater the curvature of albumin membrane vessels in diabetic adolescents, even if the urinary albumin is normal. It shows that the observation of geometric parameters of albumin membrane vessels can help to identify high-risk patients before clinical complications occur in adolescent patients with type 1 diabetes.

RETRACTED

As shown in Figure 9, after the follow-up of patients with type 2 diabetes, the OR value was 2.08, indicating that the larger the diameter of the albumin membrane vein, the easier it is to progress to DN. In addition, the diameter of albumin membrane vessels in patients with type 1 diabetes mellitus is associated with glomerular mesangial matrix hyperplasia and tubulointerstitial lesions in the early stage of DN. However, the mechanism of the relationship between the increase of albumin membrane vascular diameter and nephropathy in diabetic patients is still unclear, which may be related to tissue hypoxia and inflammation. Most of the previous studies focused on the relationship between the change of albumin membrane vascular diameter and the progression of nephropathy, and there is a lack of research on the diagnostic value of albumin membrane vascular diameter for DN. Therefore, exploring the internal relationship between albumin membrane vascular diameter and DN and providing a theoretical basis for the diagnosis of DN will become the focus of future research.

## 5. Conclusions

Before the obvious pathological changes of DKD, the whole proteome of patients has changed. Therefore, the detection and discovery of urinary microalbumin are of great significance for the early diagnosis of DKD. Urine and blood samples are convenient, safe, painless, and noninvasive and have been widely used in clinical biomarker screening. At present, DKD proteomics research mainly screens and identifies protein biomarkers from patients' urine, serum, and other noninvasive samples, in order to achieve the early diagnosis of DKD. The objective is to study the biomarkers of DKD urinary proteome. In kidney-related diseases, urine is a potential source of kidney-related biomarkers. Urine proteomics studies are an important way to investigate the associated changes in renal dysfunction. Urine protein is composed of a mixture of plasma and kidney protein, of which about 30% is plasma protein and the remaining 70% is produced in the kidney. Because the normal urine protein usually reflects the normal physiological characteristics of renal tubules, the changes of urine protein excretion can reveal the response of renal tissues such as renal tubules and glomeruli to physiological stimulation.

RETRACTED

So far, many studies have identified candidate biomarkers in urine proteome for early diagnosis and prediction of DKD progression, mainly including biomarkers reflecting renal injury caused by glomerular injury, podocyte injury, renal tubular injury, oxidative stress, inflammation, and activation of the renin-angiotensin system (RAS), such as transferrin related to glomerular injury protein, type IV collagen (IV), podx protein (podxl), and wilmstumor-1 factor related to podocyte injury.

Methods based on computational analysis and interaction model construction are gradually developed, such as gene proximity method, gene cluster method, phylogenetic spectrum, network integration, and GO-based association method. The combination of experimental methods and computational methods has further improved the quality and quantity of protein-protein interaction data. At the same time, through the collection and collation of massive data, many different protein interaction retrieval databases have been formed, such as biogrid database, dip database, MIPs database, and mint database. In the process of DKD disease development, complex biological processes involve the interaction and regulation of a variety of proteins. However, the interaction relationship between the existing candidate DKD markers has not been fully explored, which hinders the comprehensive construction of the DKD protein molecular regulatory network. This enables researchers to improve the overall interaction level through experiments and computer simulation. Therefore, it is helpful to elucidate the molecular mechanism of DKD. We have continuously improved the research system of DKD proteomics, which has laid a good technical foundation for the follow-up study of DKD pathogenesis, early diagnostic markers, therapeutic targets, and efficacy evaluation from the level of proteomics.

## Figures and Tables

**Figure 1:** Deep learning neural network model on the same data set.

**Figure 2:** The important role of removing albumin status in improving MA.

**Figure 3:** Urine microalbumin detection and analysis results.

**Figure 4:** Connecting parties in the securities market.

**Figure 5:** PDR diagnosis of DN is highly specific.

RETRACTED

**Figure 6:** Multiple mechanisms are involved in the development.

**Figure 7:** Large number of feature maps produced by convolutional neural networks.

**Figure 8:** Individual characteristics of different companies exist.

**Figure 9:** Early glomerular mesangial matrix proliferation.

**Table 1:** An increase in the depth of the network model will lead to an increase.

Item	FPG	2hPPG	HbA1c	MAU	DKD	HG
LeNet	2.33	2.93	3.53	3.68	1.47	2.74
DetectionNet	5.94	3.67	5.59	2.53	3.73	2.94
Inception	5.45	1.4	3.73	4.4	3.04	1.14
ROS	4.93	2.19	3.19	4.19	4.66	4.61
CE-MS	3.13	4.04	4.95	6.76	6.43	2.88
IV	4.81	1.87	4.91	4.77	1.58	6.86

**Table 2:** Diagnosis of diabetic albumin disease grade.

Item	MA	MAU	LeNet	DetectionNet	Inception	ROS
Gender	2.35	4.49	2.67	3.89	2.04	5.76
FPG	2.01	2.58	2.99	1.21	2.6	2.62
2hPPG	3.4	1.44	4.02	4.26	1.6	4.45
HbA1c	2.36	5.28	4.25	4.13	3.29	3.34
Age	4.78	3.22	6.75	1.29	6.14	1.96
DKD	1.11	4.9	3.92	3.44	1.03	1.81

**Table 3:** Aging-related peptide excretion patterns.

Item	2hPPG	MAU	LeNet	DetectionNet	Inception	ROS
The elderly	1.55	1.36	1.69	1.95	1.86	1.24
DKD	1.76	3.1	3.01	1.99	2.4	2.83
Biomarkers	3.08	4.55	3.25	2.07	4.91	5.33
Excretion	5.56	1.06	2.59	3.16	5.24	3.7
Gender	3.72	1.06	3.45	4.92	4.25	1.34
FPG	1.63	3.31	6.58	2.83	2.98	1.49

**Table 4:** Integrate the targeting function of proteomic network analysis.

Item	2hPPG	MAU	LeNet	DetectionNet	Inception	ROS
Protein	0.27	1.65	0.13	0.56	0.01	0.8
DKD	2.89	1.95	3.71	1.89	1.43	1.59
Biomarkers	4.76	2.34	3.01	2.29	4.7	5.15
Excretion	1.06	4.43	3	5.24	5.12	3.74
Gender	3.84	2.72	4.31	4.07	1.44	2.92
FPG	3.22	1.02	1.13	5.14	4.41	5.13

**Table 5:** Diabetic teenagers even if urine albumin is normal.

Item	ROS	MAU	LeNet	DetectionNet	Inception	2hPPG
Protein	2.4	1.27	1.75	3.11	1.58	2.19
DKD	2.34	4.55	3.83	2.55	2.97	3.6
Biomarkers	1.65	2.34	4.28	1.79	2.66	2.55
Excretion	1.89	3.38	1.73	1	1.29	3.84
Gender	2.67	1.22	5.85	6.44	4.28	6.87
FPG	5.18	1.83	3.95	1.52	2.18	4.22

## Data Availability

No data were used to support this study.

## References

[1] Shankar K., Zhang Y., Liu Y., Wu L., Chen C.-H. (2020). Hyperparameter tuning deep learning for diabetic retinopathy fundus image classification. *IEEE Access*.

[2] Knobel D. (2019). The presence and consequence of nonalbuminuric chronic kidney disease in patients with type 1 diabetes. *Preventive Veterinary Medicine*.

[3] Mise K., Hoshino J., Ueno T. (2020). Clinical and pathological predictors of estimated GFR decline in patients with type 2 diabetes and overt proteinuric diabetic nephropathy. *Diabetes Metabolism Research and Reviews*.

[4] An Y., Xu F., Le W. (2020). Renal histologic changes and the outcome in patients with diabetic nephropathy. *Nephrology, Dialysis, Transplantation: Official Publication of the European Dialysis and Transplant Association-European Renal Association*.

RETRACTED

[5] Kimura K. (2020). Clinical significance of urinary liver-type fatty acid-binding protein in diabetic nephropathy of type 2 diabetic patients. *The American Journal of Pathology*.

[6] Elhoseny M., Shankar K., Uthayakumar J. (2019). Intelligent diagnostic prediction and classification system for chronic kidney disease. *Scientific Reports*.

[7] Maratos-Flier E. (2020). Clinical significance of urinary liver-type fatty acid binding protein at various stages of nephropathy. *Annual Review of Physiology*.

[8] Groop P. H. (2020). Clinical value of NGAL, L-FABP and albuminuria in predicting GFR decline in type 2 diabetes mellitus patients. *Diabetes Care*.

[9] Hwang S. (2017). Tissue expression of tubular injury markers is associated with renal function decline in diabetic nephropathy. *Journal of Diabetes and its Complications*.

[10] Dantas R. T., Sampaio T. L., Lima D. B. (2018). Evaluation of KIM-1 as an early biomarker of snakebite-induced AKI in mice. *Toxicon*.

[11] Lippi I., Perondi F., Meucci V., Bruno B., Gazzano V., Guidi G. (2018). Clinical utility of urine kidney injury molecule-1 (KIM-1) and gamma-glutamyl transferase (GGT) in the diagnosis of canine acute kidney injury. *Veterinary Research Communications*.

[12] Viswanathan G. (2020). Tubular markers do not predict the decline in glomerular filtration rate in type 1 diabetic patients with overt nephropathy. *International Journal of Nephrology*.

[13] Poizat C. (2016). Urinary kidney injury molecule-1 and neutrophil gelatinase-associated lipocalin as indicators of tubular damage in normoalbuminuric patients with type 2 diabetes. *The Journal of Pharmacy and Pharmacology*.

[14] Tiwari S. (2020). Regression of microalbuminuria in type 1 diabetes is associated with lower levels of urinary tubular injury biomarkers, kidney injury molecule-1, and N-acetyl-beta D glucosaminidase. *PloS One*.

[15] Veron D. (2020). Kidney injury molecule-1 and the loss of kidney function in diabetic nephropathy: a likely causal link in patients with type 1 diabetes. *Nefrologia: publicacion oficial de la Sociedad Espanola Nefrologia.*.

[16] Cha D. R. (2020). Parallel increase in urinary excretion rates of immunoglobulin G, ceruloplasmin, transferrin, and orosomucoid in normoalbuminuric type 2 diabetic patients. *Diabetic Medicine: A Journal of the British Diabetic Association*.

[17] Quattrocchio G., Roccatello D. (2016). IgG4-related nephropathy. *Journal of Nephrology*.

[18] Wang K. (2018). Urinary IgG4 and Smad1 are specific biomarkers for renal structural and functional changes in early stages of diabetic nephropathy. *Kidney International Reports*.

RETRACTED

[19] Wang M. (2018). Urinary exosomal mRNA of WT1 as diagnostic and prognostic biomarker for diabetic nephropathy. *Molecular Medicine Reports*.

[20] Starczynowski D. T. (2020). Wilm’s tumor-1 protein levels in urinary exosomes from diabetic patients with or without proteinuria. *Oncotarget*.

[21] Zhang Y., Chen X., Yuan L. (2018). Down-regulation of IRAK1 attenuates podocyte apoptosis in diabetic nephropathy through PI3K/Akt signaling pathway. *Biochemical and Biophysical Research Communications*.

[22] Fasshauer M. (2020). IRAK1: oncotarget in MDS and AML. *Clinical Endocrinology*.

[23] Kimura K. (2020). Urinary liver-type fatty acid-binding protein and progression of diabetic nephropathy in type 1 diabetes. *Clinica Chimica Acta; International Journal of Clinical Chemistry*.

[24] Moresco R. N. (2020). Using participatory epidemiology to investigate management options and relative importance of tick-borne diseases amongst transhumant zebu cattle in Karamoja Region, Uganda. *Clinical Biochemistry*.

[25] Forsblom C. M. (2020). Heat shock protein 72 (Hsp72) specific induction and temporal stability in urine samples as a reliable biomarker of acute kidney injury (AKI). *Diabetes Care*.

[26] Liu R. (2017). NLRP3 expression and urinary HSP72 in relation to biomarkers of inflammation and oxidative stress in diabetic nephropathy patients. *Journal of Clinical Laboratory Analysis*.

[27] Ma Y. (2019). Diabetic kidney disease: a clinical update from kidney disease: improving global outcomes. *International Journal of Clinical and Experimental Pathology*.

[28] Li C., Liu P., Zou C., Sun F., Cioffi J. M., Yang L. (2015). Spectral-efficient cellular communications with coexistent one-and two-hop transmissions. *IEEE Transactions on Vehicular Technology*.

[29] Chen Y., Zheng W., Li W., Huang Y. (2021). Large group Activity security risk assessment and risk early warning based on random forest algorithm. *Pattern Recognition Letters*.

[30] Elhoseny M., Shankar K. (2019). Optimal bilateral filter and convolutional neural network based denoising method of medical image measurements. *Measurement*.

